# CPE Regulates Proliferation and Apoptosis of Primary Myocardial Cells Mediated by Ischemia and Hypoxia Injury

**DOI:** 10.1155/2022/3155171

**Published:** 2022-03-16

**Authors:** Jin Li, Zishuang Dong, Yuxiong Pan, Luchen Wang, Wei Zhao, Jian Zhang

**Affiliations:** ^1^Department of Cardiology, The Affiliated Longyan First Hospital of Fujian Medical University, Longyan, Fujian 364000, China; ^2^Department of Cardiology, Xuzhou Central Hospital, Xuzhou, Jiangsu 221000, China; ^3^Department of Cardiovascular Surgery, Fuwai Hospital, National Center for Cardiovascular Diseases, Chinese Academy of Medical Sciences, Peking Union Medical College, Beijing 100037, China; ^4^Division of Cardiology, The First Affiliated Hospital with Nanjing Medical University, Nanjing 210000, China

## Abstract

**Objective:**

To observe the effect of carboxypeptidase E (CPE) on the ischemia and hypoxia (I/H) injury of primary cardiomyocytes.

**Methods:**

Quantitative real-time polymerase chain reaction (qRT-PCR) technology was used to detect the expression of CPE in sham and myocardial infarction (MI) rat heart tissue, and the plasmid was transferred into primary cardiomyocytes by transfection technology. The apoptosis rate of cardiomyocytes was detected by terminal deoxynucleotidyl transferase-mediated dUTP-biotin nick end labeling (TUNEL) staining, Annexin V-PI staining, and Cell Counting Kit-8 (CCK-8) assay. In addition, Caspase kit and qRT-PCR technology were used to detect the expression of apoptosis-related factors. The cell proliferation was detected by 5-ethynyl-2'-deoxyuridine (EdU) staining, flow cytometry, and qRT-PCR technology. In addition, Western blotting (WB) and qRT-PCR techniques were used to detect the Wnt/*β*-catenin pathway.

**Results:**

First, we found that the expression of CPE in the marginal zone of MI was obviously reduced. Overexpression of CPE in primary cardiomyocytes can effectively inhibit ischemia/hypoxia (I/H)-induced apoptosis and decreased cell activity. In addition, CPE can promote cell proliferation and relieve the inhibitory effect of I/H on cardiomyocytes. At the same time, CPE can promote the expression of *β*-catenin and c-myc.

**Conclusion:**

Overexpression of CPE in primary cardiomyocytes can effectively alleviate the decreased cell activity, increased apoptosis, and decreased proliferation caused by I/H and regulated by Wnt/*β*-catenin pathway.

## 1. Introduction

Acute myocardial infarction (AMI) is a disease with high morbidity and mortality worldwide and is the most common cause of heart failure (HF). Recent epidemiological investigations show that the incidence of AMI is increasing year by year and that it has become a cardiovascular emergency that seriously endangers the life and health of middle-aged and elderly people [1]. The main pathophysiological mechanism of MI is the rupture of coronary atherosclerotic plaque, which causes thrombotic obstruction. After MI, the left ventricle undergoes changes from molecules to cells to extracellular matrix, which obviously changes its size, shape, and function at the organ level. The left ventricle expands progressively and decreases its contractile function, eventually leading to HF and death [2, 3]. Although heart transplantation is the most effective way to treat end-stage HF and restore cardiac function, limited donors are far from being able to meet the needs of patients with HF whose morbidity is gradually increasing, and transplant patients need to take long-term immunosuppressants after transplantation. Because of multiple problems such as infection and immune rejection, only a few patients can benefit from it [4]. Therefore, to find an effective treatment strategy to promote myocardial cell proliferation and reverse myocardial cell loss after MI has always been a research hotspot.

Carboxypeptidase (CP) is an exopeptidase that specifically degrades and releases free amino acids from the C-terminus of the peptide chain one by one. At present, different kinds of CP have been proved to be involved in cell proliferation, cell differentiation, cell cycle, and cell apoptosis [5, 6]. Zaninotto et al.'s study found that CPN reached its peak at 48 hours in patients with AMI [7]. In addition, Anta Ngkelo also confirmed that CPA can reduce HF caused by MI [8]. In addition, CPE has been shown to be a multifunctional protein, which plays an important role in regulating the balance of endocrine and nervous system, as well as the occurrence of coronary heart disease (CHD) [9, 10]. However, there are few studies on its role in MI. Therefore, we assume that CPE gene may be closely related to the occurrence and prognosis of MI.

The relationship between Wnt signaling pathway and MI is one of the hotspots in the research on the pathological mechanism of MI in recent years. Wnt signaling pathway not only participates in the key process of heart development, but also plays a crucial role in various pathological processes such as MI, myocardial hypertrophy, myocardial fibrosis, and HF after adulthood [11, 12]. Among them, Wnt3a can promote the proliferation and differentiation of embryonic stem cells and also plays a crucial role in the development and differentiation of cardiomyocytes [13]. Moreover, in the process of HF, studies have shown that Wnt3a can regulate the proliferation of cardiomyocytes through Dapper-1 regulating *β*-catenin signaling pathway [14]. Therefore, we speculated whether CPE could also regulate myocardial cell apoptosis and proliferation reduction induced by MI through Wnt/*β*-catenin pathway.

## 2. Materials and Method

### 2.1. Experimental Animals and Model Preparation

Twenty-four 8-week-old male Sprague Dawley rats, weighing 200–250 g, were purchased from Beijing Weitong Lihua Experimental Animal Technology Co. They were randomly divided into sham operation group (sham group, *n* = 12) and acute myocardial infarction group (MI group, *n* = 12). The rats were anesthetized by intraperitoneal injection of 3% pentobarbital sodium, and the small animal ventilator was connected after tracheal intubation. Subsequently, the left atrial appendage and left ventricle were fully exposed, and the open-heart pericardium was torn. A noninvasive small round needle was inserted into the lower edge of the left atrial appendage 2-3 mm with a silk thread, passing through the surface of the myocardium under the left descending coronary artery and then ligated. The obvious elevation of the ST segment of the electrocardiogram was a sign of successful ligation. The procedures of tracheal intubation, thoracotomy, and anterior descending branch suture in the sham group were the same as those in the MI group, but the left coronary artery was not ligated.

### 2.2. Echocardiography

We used GE Vivid 7 ultrasonic diagnostic apparatus, with probe frequency of 12 MHz, to perform echocardiography in rats and recorded left ventricular end-diastolic diameter (LVEDD), left ventricular end-systolic diameter (LVESD), ventricular end-diastolic volume (EDV), and ventricular end-systolic volume (ES). The left ventricular fractional shortening (FS)% = (LVEDD − LVESD)/LVEDD* *×* *100%; the left ventricular ejection fraction (EF)% = (EDV − ES)/EDV* *×* *100%.

### 2.3. Hematoxylin-Eosin (H&E) Staining

After the tissue sections were dewaxed and hydrated, the H&E staining solution was prepared according to the instructions. After sealing, the slices were observed under a light microscope and photographed.

### 2.4. Lactate Dehydrogenase (LDH) Activity

On the second day after surgery, blood was collected from orbital venous plexus of rats. 10 *μ*L of rat serum from each group was taken, and 10 *μ*L of cell lysis buffer was added for lysis. Then, LDH detection kit (Jiancheng, Nanjing, China) was used to detect LDH activity, and LDH enzyme activity was calculated according to the standard curve.

### 2.5. Primary Cardiomyocyte Extraction

The newborn SD rats' hearts were taken out under aseptic conditions after sterilization, and excess tissues were removed. Then, the ventricle was cut into tissue pieces of about 1 mm^3^ uniform size, and 0.125% Trypsin (Elabscience, Wuhan, China) was used to digest the tissue 4 times, 10 minutes each. The digested cell suspension was absorbed into the centrifuge tube, and Dulbecco's Modified Eagle's Medium (DMEM; Life Technology, Wuhan, China) medium containing 10% fetal bovine serum (FBS; Life Technology, Wuhan, China) was added to terminate digestion. After centrifugation, the supernatant was discarded, and the cell suspension was resuspended to complete medium and was uniformly inoculated in an incubator at 37°C. Fibroblasts were removed by differential adherent method, and the cardiomyocytes were inoculated on the culture plate after adjusting the cell concentration. The cardiomyocytes were further cultured in the cell incubator, and the experiment was carried out after incubation for 36 hours.

### 2.6. Transfection

The primary cardiomyocytes were seeded into a 6-well cell culture plate at a density of 1 × 10^5^ cardiomyocytes per well, and then the cardiomyocytes were allowed to place overnight in incubator. Using Lipofectamine^TM^ 3000 (Rib Bio, Guangzhou, China) as a vector, the overexpression plasmid CPE (pcDNA3.1-CPE) and its negative control plasmid (pcDNA3.1) were transfected into the cardiomyocytes according to the dosage and method in the instructions, and then the complete medium was changed after static culture for 6 hours to stop transfection. After culturing for 36 hours, the cardiomyocytes were collected and tested for transfection efficiency.

### 2.7. Cell Processing

48 hours after the transfection, the low-sugar DMEM medium without FBS was replaced to simulate the ischemic state. At the same time, the cardiomyocytes were placed in a hypoxic tank, which was placed in a 37°C-cell incubator. After the oxygen concentration in the hypoxia culture tank drops to about 0.1%, the hypoxia time will be calculated. This experiment took ischemia/hypoxia (I/H) 8 hours as the intervention time point.

### 2.8. Terminal Deoxynucleotidyl Transferase-Mediated dUTP-Biotin Nick End Labeling (TUNEL) Staining

The transfected primary cardiomyocytes were inoculated in a 12-well plate, and the cell density was controlled to about 70%. Subsequently, the primary cardiomyocytes were treated differently. After 8 hours, the cardiomyocytes were washed with precooled phosphate buffered saline (PBS) solution 2 times, 5 minutes each; 4% paraformaldehyde was used to fix the cardiomyocytes for 20 minutes; and the cardiomyocytes were incubated with 0.5% Triton X-100 (Sinopharm Chemical Reagent, Shanghai, China) at room temperature for 10 minutes. After washing the cardiomyocytes with PBS 3 times, each well was incubated with TUNEL reagent (Gene, Shanghai, China) at 37°C for 1 hour. After washing the cardiomyocytes with PBS, the nucleus was stained with DAPI reagent, and the positive cells were observed under an inverted fluorescence microscope (Thermo Fisher Scientific, Waltham, MA, USA). ImageJ software was used to exclude false positives and count EdU positive cells.

### 2.9. Cell Counting Kit-8 (CCK8) Assay

Each group of primary cardiomyocytes was randomly selected, CCK-8 reagent (Ye Sen, Shanghai, China) was added to each well of the medium in a ratio of 10 : 1, the 96-well plate was cultured in an incubator at 37°C for 2 hours in the dark, and the optical density (OD) was measured with a microplate reader at 450 nm wavelength. The OD value indirectly reflects the viability of cardiomyocytes, and the cell viability (%) was calculated according to the instructions.

### 2.10. Caspase-3 and Caspase-9 Activity Detection

Caspase-3 and Caspase-9 activity assay kits (Jiancheng, Nanjing, China) were used, and the operation was performed in accordance with the instructions. The activity change was expressed by the absorbance of the microplate reader (Thermo Fisher Scientific, Waltham, MA, USA) at a wavelength of 405 nm.

### 2.11. Cell Cycle Detection

Primary cardiomyocytes were inoculated in a 6-well plate, and cell treatment was performed as described above. After 8 hours of treatment, the cardiomyocytes were collected and fixed with prechilled 75% ethanol. Subsequently, the collected primary cardiomyocytes were processed in accordance with the operating instructions of the cell cycle kit (Gene, Shanghai, China), treated at room temperature, protected from light for 30 minutes, and then detected by flow cytometry. The collected data was processed and analyzed by the instrument software.

### 2.12. Apoptosis Detection

The primary cardiomyocytes of each group were collected, and the collected cardiomyocytes were processed according to the Annexin V-PI cell apoptosis kit (Gene, Shanghai, China) operating instructions, reacted for 15 minutes at room temperature in the dark, and then were detected by flow cytometry. The collected data was processed and analyzed by the FlowJo v10 software.

### 2.13. Western Blotting Technology

The protein was extracted with protein lysate containing 1% PMSF (Thermo Fisher Scientific, Waltham, MA, USA), and the protein content of each group was detected according to the requirements of the bicinchoninic acid (BCA) protein kit (R&D Systems, Minnesota, USA). Sodium dodecyl sulphate-polyacrylamide gel electrophoresis (SDS-PAGE) gel was used for protein electrophoresis, and then the transfer reaction was performed after blocking the polyvinylidene difluoride (PVDF; Thermo Fisher Scientific, Waltham, MA, USA) membrane with 5% skim milk for 2 hours. The primary antibody (*β*-catenin, Abcam, Cambridge, MA, USA, Rabbit, 1 : 2000; p-*β*-catenin, Abcam, Cambridge, MA, USA, Rabbit, 1 : 1000; GAPDH, Proteintech, Rosemont, USA, 1 : 2000) was added and incubated overnight at 4°C. The next day, the membrane was immersed in the secondary antibody (Abcam, Cambridge, MA, USA, 1 : 2000) and incubated for 1 hour. After washing the membrane, enhanced chemiluminescence (ECL, Yifei Xue Biotechnology, Nanjing, China) technology was used for luminescence development. With GAPDH as an internal reference, ImageJ software was used to quantitatively analyze protein expression.

### 2.14. Quantitative Real-Time Polymerase Chain Reaction (qRT-PCR)

Rat myocardial tissue and primary cardiomyocytes total RNA were extracted by Trizol reagent (Thermo Fisher Scientific, Waltham, MA, USA), the eligible RNA was reverse-transcribed into cDNA, and then fluorescence quantitative PCR amplification was performed. Reaction conditions were as follows: predenaturation at 95°C for 10 minutes, 1 cycle; denaturation at 95°C for 15 seconds; annealing at 60°C for 30 seconds; extension at 72°C for 30 seconds, a total of 38 cycles. Using GAPDH as an internal control, the relative expression of each gene was expressed as 2^−△△CT^. Primers used are shown in Table 1.

### 2.15. 5-Ethynyl-2'-deoxyuridine (EdU) Staining

The transfected primary cardiomyocytes were inoculated in a 24-well plate, and the cell density was controlled to about 70%. Then, the cardiomyocytes were grouped and processed for 8 hours. According to the instructions of the EdU kit (Gene, Shanghai, China), 10 *μ*mol/L EdU reagent was added to each well, and after incubation for 2 hours, the reagent that did not penetrate DNA was washed away by PBS. 4% paraformaldehyde was used to fix the cardiomyocytes for 20 minutes. After washing with PBS, Apollo staining solution was added to each well and incubated in the dark at room temperature for 30 minutes. After washing the staining solution with PBS, DAPI reagent was used to stain the nucleus for 5 minutes. The image was observed under a fluorescence microscope, and ImageJ software was used to exclude false positives and count EdU positive cells.

### 2.16. Statistical Analysis

SPSS 21.0 software was used for data processing and statistical analysis. The measurement data were expressed as mean ± standard deviation (*X *±* *SD). One-way ANOVA was used to deal with the mean comparison between groups. SNK-q test was used to deal with pairwise comparison between groups. *P* < 0.05 indicated that the difference was statistically significant.

## 3. Results

### 3.1. Damage to the Structure and Function of the Rat Heart after MI

Compared with the sham group, the LDH activity in the serum of the MI group increased obviously after two days of MI surgery (Figure 1(a)). Next, in the second and fourth weeks after the operation, the H&E staining results indicated that the myocardial structure of the MI group was disordered in the second week after MI. Inflammatory cells in the interstitial space were infiltrated by normal muscle tissue and replaced by fibrous tissue. In the fourth week, the myocardial structure was still disordered (Figure 1(b)). At the same time, the echocardiographic results indicated that the cardiac function of the MI group was obviously impaired; the LVEF% and LVFS% were obviously reduced in the second and fourth weeks after MI (Figures 1(c) and 1(d)). All the above results show that our model construction was successful. Then, the collected tissues were subjected to qRT-PCR detection, and the results confirmed that the CPE expression in the marginal area of MI was obviously reduced (Figure 1(e)).

### 3.2. Overexpression of CPE Can Inhibit I/H-Induced Apoptosis of Primary Cardiomyocytes

First, we collected cardiomyocytes from the control group and the I/H group for qRT-PCR detection. The results showed that the CPE expression of primary cardiomyocytes was obviously reduced after I/H treatment, which was consistent with the results of in vivo experiments (Figure 2(a)). Therefore, we transfected pcDNA3.1-CPE and pcDNA3.1 into cardiomyocytes and used qRT-PCR experiments to verify the transfection efficiency (Figure 2(b)). Then, TUNEL staining was used to detect the four groups of cardiomyocytes. The results indicated that the number of TUNEL-positive cells in the I/H was obviously more than that in the control group. In the I/H + pcDNA3.1-CPE group, the number of TUNEL-positive cells was obviously reduced (Figure 2(c)). At the same time, similar results were obtained in the detection of apoptosis level by flow cytometry (Figure 2(d)). Secondly, compared with the control group, the cell activity of the I/H group was obviously reduced, while the cell activity of the I/H + pcDNA3.1-CPE group was obviously increased (Figure 2(e)). In addition, the activities of Caspase-3 and Caspase-9 in the cell supernatant of the I/H group were also obviously increased. On the contrary, when the primary cardiomyocytes overexpressed CPE, the activities of Caspase-3 and Caspase-9 in the cell supernatant were obviously reduced (Figures 2(f) and 2(g)). Furthermore, the qRT-PCR results indicated that the expression of Bax increased after the cardiomyocytes were treated with I/H, and the expression of Bcl-2 decreased. However, after the primary cardiomyocytes overexpressed CPE, we obtained the opposite result (Figures 2(h) and 2(i)).

### 3.3. Overexpression of CPE Can Inhibit the Reduction of Primary Cardiomyocyte Proliferation Caused by I/H

Then, the immunofluorescence technology was used to detect the proliferation of the 2 groups of cardiomyocytes. EdU is effective indicators for detecting cell proliferation. The staining results showed that, compared with the pcDNA3.1-NC group, the rate of EdU positive cells in the pcDNA3.1-CPE group was obviously increased, indicating that CPE could promote cell proliferation (Figure 3(a)). Then, flow cytometry was used to detect the four groups of cell cycles, showing that the I/H group cardiomyocytes accumulated in *G*0 + *G*1 phase, the number of S phase cardiomyocytes was small, and the number of S phase cardiomyocytes of I/H + pcDNA3.1-CPE group increased obviously (Figure 3(b)). At the same time, qRT-PCR detection of cycle-related factors cyclin D1 and cyclin-dependent kinase 4 (CDK4) showed that, compared with the control group, the expression of cyclin D1 and CDK4 in the I/H group was obviously reduced, while the expression of cyclin D1 and CDK4 was obviously increased in the I/H + pcDNA3.1-CPE group (Figures 3(c) and 3(d)).

### 3.4. Overexpression of CPE Can Activate Wnt/*β*-Catenin Signaling Pathway

In order to detect the effect of Wnt/*β*-catenin signaling pathway in the I/H process of primary cardiomyocytes and the role of CPE, we first detected the protein expression of *β*-catenin and p-*β*-catenin in the four groups of cardiomyocytes. The results showed that the expression of *β*-catenin was decreased and the expression of p-*β*-catenin was increased in I/H group. Compared with the I/H group, the *β*-catenin expression in the I/H + pcDNA3.1-CPE group was relatively higher, and the p-*β*-catenin expression was relatively lower (Figure 4(a)). Next, qRT-PCR was used to detect *β*-catenin and c-myc expression. The results indicated that the mRNA expression of *β*-catenin and c-myc decreased in the I/H group, while the mRNA expression in the I/H + pcDNA3.1-CPE group was upregulated obviously (Figures 4(b) and 4(c)).

## 4. Discussion

The small animal MI model is currently one of the best models for studying cardiomyocyte apoptosis and ventricular remodeling after MI and is widely recognized and applied. This model permanently blocks the blood supply of the ligated distal myocardium by ligating the anterior descending branch, and the distal cardiomyocyte ischemia and hypoxia eventually undergo apoptosis. In this study, the rat MI model was used to simulate the pathological model of clinical MI patients. We successfully established a rat MI model. After MI operation, the serum LDH content was obviously increased, and histology also confirmed the presence of fibrosis and inflammatory cell infiltration in the infarct area. At the same time, cardiac function was significantly reduced in the MI group at the second and fourth weeks.

CPE is a member of the M14 family of metal carboxypeptidases and is the most important carboxypeptidase in the biosynthesis of a variety of hormone peptides and neurotransmitters. Studies have found that CPE is one of the important enzymes in the process of enzymatic hydrolysis of proinsulin into insulin and C-peptide, and epidemiological statistics show that high proinsulin levels are an independent risk factor for CHD. Therefore, the change of CPE gene must be closely related to the development of CHD. Then, we assume that CPE plays a crucial role in the process of MI. In our research, we found that CPE expression was decreased in the model group, which was consistent with our prediction.

A large number of studies have confirmed that the GSK3*β*/*β*-catenin signaling pathway is involved in the regulation of myocardial ischemia and hypoxia injury [15, 16]. CircSNRK was confirmed to protect against ischemia-hypoxia-induced myocardial injury by upregulating *β*-catenin expression and inhibiting *β*-catenin phosphorylation [17]. Studies have found that Wnt protein binds to Frizzled (FZD) heterodimeric receptor and low-density lipoprotein receptor-related protein 5/6 (LRP5/6). When the FZD/LRP receptor is not bound, glycogen synthase kinase-3*β* (GSK-3*β*) and Casein kinase 1 (CK1) gradually phosphorylate *β*-catenin, causing it to be ubiquitinated and decomposed by some proteasomes. When Wnt protein binds to FZD and LRP, the complex loses its effect. Therefore, the dephosphorylation of *β*-catenin in the cytoplasm makes it accumulate in the cytoplasm and transfer to the nucleus when it reaches a certain concentration, and it binds to the T cell transcription factor/lymphoid enhancer factor (TCF/LEF) in the nucleus [18]. The combination of the two will promote the transcription of related target genes, such as c-myc and cyclin D1 [19]. Similarly, our results also found that *β*-catenin expression in cardiomyocytes of I/H group was changed and *β*-catenin phosphorylation was upregulated. The difference was that the expression of *β*-catenin increased in the I/H + pcDNA3.1-CPE group, and its phosphorylation was inhibited. qRT-PCR detection of downstream c-myc transcription level found that its expression level was inhibited in the I/H group but increased in the I/H + pcDNA3.1-CPE group. This suggested that the Wnt/*β*-catenin signaling pathway was involved in the CPE-mediated I/H process of cardiomyocytes.

After MI, cardiomyocytes are ischemic and hypoxic and soon begin to apoptosis. Therefore, we simulated this process with primary cardiomyocytes in vitro. After the primary cardiomyocytes were treated with I/H, the cell viability was obviously reduced, and the cardiomyocytes were apoptotic. The number of TUNEL-positive cells increased, and the apoptosis rate of Annexin V-PI stained cells increased. There are two main apoptosis pathways, namely, death receptor (exogenous) pathway and mitochondrial (endogenous) pathway. Both can eventually lead to the activation of Caspase, which is an enzyme family that acts as a death effector molecule in various forms of cell death. Caspase-3 and Caspase-9 are important effector enzymes in the family [20]. We tested the above-mentioned enzymes in the cell culture medium and found that after the cardiomyocytes were treated with I/H, the activities of both were obviously increased, and when the cardiomyocytes overexpressed CPE, the activities of both were effectively inhibited. In addition, the Bcl-2 family is usually divided into antiapoptotic and proapoptotic members, which are differentially regulated but have similar structural homology [21]. qRT-PCR results showed that CPE can inhibit I/H-induced increase in apoptosis gene Bax and decrease in antiapoptotic gene Bcl-2. The above results suggested that the cardiomyocyte apoptosis induced by I/H can be regulated by CPE.

In normal cells, the maintenance of the cell cycle is strictly controlled by monitoring proteins including cyclin and CDK. When the cell receives the mitosis signal, the cell exits G0 stage and enters G1 stage. Subsequently, cyclin D binds to CDK4 and CDK6, resulting in partial inactivation of the Rb family of proteins, allowing the cell to enter the S phase. Cyclin A then binds to CDK1, causing cells to begin dividing [22, 23]. At the same time, we found that after cardiomyocytes overexpressed CPE, the positive cell of EdU was higher than that of I/H group. In addition, the cell cycle test results also confirmed our speculation that CEP can promote cardiomyocytes to enter S phase. The qRT-PCR results also showed that CPE can inhibit the downregulation of cyclin D1 and CDK4 induced by I/H. The above results confirmed that overexpression of CPE can regulate the proliferation cycle of cardiomyocytes.

Based on the above results, we believe that CPE can be involved in the regulation of cell cycle and apoptosis of cardiomyocytes after I/H injury through the Wnt/*β*-catenin pathway.

## 5. Conclusion

CPE regulates the decrease in the activity and proliferation of primary cardiomyocytes and the increase in apoptosis caused by I/H injury through the Wnt/*β*-catenin pathway. This will provide a new target for the treatment of MI.

## Figures and Tables

**Figure 1:** Damage to the structure and function of the rat heart after MI. (a) The serum LDH content of rats after two days of MI surgery. (b) H&E staining performed for rat hearts after two weeks or four weeks of MI surgery. (c) The cardiac function LVEF% of rats after two weeks or four weeks of MI surgery. (d) The cardiac function LVFS% of rats after two weeks or four weeks of MI surgery. (e) CPE mRNA expression in rat heart tissue after two weeks or four weeks of MI surgery. (Sham, MI-14-day, and MI-28-day groups.) ^*∗*^*P* < 0.05, compared with sham-14-day or 28-day group.

**Figure 2:** Overexpression of CPE can inhibit I/H-induced apoptosis of primary cardiomyocytes. (a) CPE mRNA expression in primary cardiomyocytes (control and I/H groups). ^*∗*^*P* < 0.05, compared with control group. (b) CPE mRNA expression in primary cardiomyocytes. (c) TUNEL staining and quantitative analysis of TUNEL-positive cells. (d) Annexin V-PI staining detection for primary myocardial cell apoptosis. (e) CCK-8 assay for the primary myocardial cell activity. (f) Caspase-3 kit to detect the content of Caspase-3 in the supernatant of primary myocardial cells. (g) Caspase-9 kit to detect the content of Caspase-9 in the supernatant of primary myocardial cells. (h) Bax mRNA expression in primary cardiomyocytes. (i) Bcl-2 mRNA expression in primary cardiomyocytes. (Control, I/H, I/H + pcDNA3.1-CPE, and I/H + pcDNA3.1 groups). ^*∗*^*P* < 0.05, compared with control group; ^#^*P* < 0.05, compared with I/H group.

**Figure 3:** Overexpression of CPE can inhibit the reduction of primary cardiomyocyte proliferation caused by I/H. (a) EdU staining and quantitative analysis of primary myocardial cells. (pcDNA3.1 and pcDNA3.1-CPE groups). ^*∗*^*P* < 0.05, compared with pcDNA3.1 group. (b) Detection of primary myocardial cell cycle by flow cytometry. (c) Cyclin D1 mRNA expression in primary cardiomyocytes. (d) CDK4 mRNA expression in primary cardiomyocytes. (Control, I/H, I/H + pcDNA3.1-CPE, and I/H + pcDNA3.1 groups). ^*∗*^*P* < 0.05, compared with control group; ^#^*P* < 0.05, compared with I/H group.

**Figure 4:** Overexpression of CPE can activate Wnt/*β*-catenin signaling pathway. (a) Protein expression and semiquantitative analysis of *β*-catenin and p-*β*-catenin in primary myocardial cells. (b) *β*-catenin mRNA expression in primary cardiomyocytes. (c) c-myc mRNA expression in primary cardiomyocytes. (Control, I/H, I/H + pcDNA3.1-CPE, and I/H + pcDNA3.1 groups). ^*∗*^*P* < 0.05, compared with control group; ^#^*P* < 0.05, compared with I/H group.

**Table 1:** qRT-PCR primers.

Gene name	Forward (5'* *>* *3')	Reverse (5'* *>* *3')
Bax	CAGTTGAAGTTGCCATCAGC	CAGTTGAAGTTACCATCAGC
Bcl-2	GACTGAGTACCTGAACCGGCATC	CTGAGCAGCGTCTTCAGAGACA
CPE	CAGCAAGAGGACGGCATCTC	GTCCAACCGCCTCATTACCAT
*β*-Catenin	GATTAACTATCAGGATGACACA	TCCATCCCTTCCTGCTTAGTC
c-myc	ATGCCCCTCAACGTGAACTTC	CGCAACATAGGATGGAGAGCA
Cyclin D1	GCGTACCCTGACACCAATCTC	CTCCTCTTCGCACTTCTGCTC
CDK4	GATTGCCTCCAGAAGACG	GGTCAGCATTTCCAGCA
GAPDH	ACAACTTTGGTATCGTGGAAGG	GCCATCACGCCACAGTTTC

RT-PCR: quantitative reverse-transcription polymerase chain reaction.

## Data Availability

The data that support the finding of this study are available from the corresponding upon reasonable request.
